# Video-Assisted Health Education Promotes Rehabilitation Training of Total Knee Arthroplasty Patients and Reduces Stress and Burnout in Nurses Compared to Oral Education

**DOI:** 10.1155/2021/5058899

**Published:** 2021-10-22

**Authors:** Ping Li, Xing Li, Hua Meng, Ling Huang, Li Zhang, Shuang Wang, Shaohua Chen

**Affiliations:** ^1^Department of Joint Surgery, Shandong Provincial Hospital Affiliated to Shandong First Medical University, Jinan 250000, China; ^2^Department of Orthopedic Surgery, The Second Affiliated Hospital of Guangzhou University of Chinese Medicine, Guangzhou 510120, China; ^3^Department of Joint Surgery/Sports Medicine, The Second Hospital, Cheeloo College of Medicine, Shandong University, Jinan 250033, China

## Abstract

Emerging evidence suggests video-assisted health education being an effective way in promoting rehabilitation. The present study was aimed at evaluating the effectiveness of video-assisted health education in promoting rehabilitation training in postoperative OA patients and at comparing it with oral education. This study was a noncontemporaneous control study involving 179 patients who underwent TKA. For the intervention group, a bedside interactive system that recorded a series of educational videos showing a rehabilitation training program was established. For the control group, oral education having the same content as that in the videos for the intervention group was provided. After education, clinical outcomes such as occurrence of complications, circulating biomarkers of inflammation, and rehabilitation progress of the patients were obtained. Furthermore, job stress and burnout in nurses who participated in the present study were assessed. Results showed that C-reactive protein levels of patients were significantly lower in the intervention group than in the control group (84.54 ± 36.09 vs. 99.45 ± 31.73 mg/L, *P* = 0.004). Faster achievement of postoperative knee flexion to 90 degrees (21.31 ± 5.83 vs. 35.72 ± 9.93 h, *P* < 0.001) and first ambulation (19.91 ± 4.57 vs. 50.15 ± 7.00 h, *P* < 0.001), reduced number of postoperative complications such as postoperative orthostatic intolerance (7 vs. 19, *P* = 0.008) and constipation (10 vs. 23, *P* = 0.009), and reduced length of hospital stay (7.51 ± 1.79 vs. 8.21 ± 2.15 days, *P* = 0.019) in the intervention group in comparison to the control group were noted. Emotional exhaustion and burnout of nurses were reduced significantly in the intervention group than in the control group (21.00 ± 8.04 vs. 36.50 ± 11.22, *P* = 0.002; 55.90 ± 11.57 vs. 85.50 ± 6.80, *P* < 0.001, respectively). Reduced personal accomplishments in nurses were improved significantly in the intervention group when compared with the control group (41.90 ± 4.91 vs. 32.80 ± 7.07, *P* = 0.004). We concluded that video-assisted health education may promote TKA patient recovery and reduce burnout and stress in nurses when compared with oral education. Video-assisted health education could be helpful in situation where manpower of nurse is in shortage.

## 1. Introduction

Knee osteoarthritis (KOA) is a chronic, progressive, and recurrent joint disorder that leads to joint instability and physical disability [1]. KOA is multifactorial in origin, and both inflammatory and biomechanical whole-organ disease processes play an important role in disease progression [2–4] that is affected by several factors, including family history, age, obesity, diabetes, and synovitis [5]. KOA has a prevalence rate of up to 8.1% with a higher frequency among women than among men at any given age more than 50 years old [5]. For patients who are at the end stage of KOA, total knee arthroplasty (TKA) has been demonstrated to be an effective treatment [6] and postoperative training after TKA is receiving growing attention from clinicians globally.

Elevated immune response was observed following TKA procedures. Increased immune response, systematic or localized, to acute oxidative stress and levels of cytokines after surgery was reported [7, 8]. Postoperative complications such as postoperative orthostatic intolerance [9] and deep vein thrombosis [10] could contribute to the stress and thus lead to a slow recovery of patients. As an antioxidant stress strategy, postoperative rehabilitation training could reduce circulating markers of neutrophil activation and the concentration of cytokines [11, 12]. In several areas around the world, such as China, the most common way of implementing postoperative rehabilitation training health education is through oral education provided by nurses, while the nurses in these areas are experiencing high workloads nowadays [13].

Recently, video-assisted health education, a fast and intuitive educational method, has been reported to be helpful for patients to understand health information and thus improve their acceptance and promote their rehabilitation [14]. Studies showed that video-assisted health education can significantly improve the quality of life in patients with bronchiectasis and reduce the complications [15]. Furthermore, video-assisted health education was suggested to be able to reduce burnout in nurses that was caused by heavy workload and could improve work efficiency and job satisfaction in nurses [16]. However, to the best of our knowledge, the current evidence is insufficient to determine the effects of video-assisted health education on rehabilitation in patients who have undergone TKA and on work stress of nurses. We hypothesized that video-assisted health education could promote postoperative recovery and reduce burnout and job stress in nurses when compared with oral education.

## 2. Materials and Methods

### 2.1. Ethics

The present study was conducted after approval by the Research Ethics Committee of Shandong Provincial Hospital affiliated to Shandong First Medical University (no. 2017-055) and was reported in accordance with the CONSORT 2010 statement. Written consent was obtained from each patient who participated in the study.

### 2.2. Participants and Baseline Information

The present study was a noncontemporaneous control study. A convenience sampling method was used for the recruitment of subjects from January 2018 to October 2019. Subjects who met the following inclusion criteria were included: (1) 18 years of age or older and (2) subjects who were diagnosed as having degenerative osteoarthritis and underwent primary TKA. The exclusion criteria were as follows: (1) having any diagnosed hip or ankle disorders, (2) having any balance disorders or ligament instability, (3) severe osteoporosis or severe cardiopulmonary diseases, or (4) ankylosing spondylitis, hemophilic arthritis, and severe deformities of the knee joint due to diseases other than KOA that could affect the results. Subjects who underwent TKA from January 2018 to December 2018 were assigned to the control group, and the patients from January 2019 to October 2019 who underwent TKA were assigned to the intervention group.

Baseline information including age, gender, marital status, and education level, comorbidities, and osteoarthritis history were obtained on the day of admission. The Numerical Rating Scale (NRS) was used to evaluate pain, and the Barthel index (BI) was used to evaluate the ability of daily living.

### 2.3. Intervention

A standardized exercise plan for TKA patients was developed by the rehabilitation team in our hospital. The content of the exercise plan included ankle pump, isometric contraction, straight leg raising, and flexion knee exercises (Table 1). A 3-minute video that showed the exercise plan was made, and a bedside interactive system was established for playing the video.

The patients in the control group were provided with oral education by the trained nurses about the exercise plan shown in Table 1. The patients in the intervention group were provided with a demonstration of the exercises (Table 1) and then were shown with the video by the bedside interactive system. The patients were quizzed to test their level of comprehension regarding the exercise plan, and tutorial was provided as needed.

### 2.4. Postoperative Recovery

The time to achieve first ambulation, straight leg elevation, and knee flexion to 90 degrees was evaluated at 8:00 am, 12:00 pm, 16:00 pm, and 22:00 pm every day. Occurrence of the following postoperative complications was recorded if they were diagnosed following the criteria reported elsewhere [17–19]: (1) deep venous thrombosis (DVT), (2) postoperative orthostatic intolerance, and (3) constipation. Venous blood samples were collected by trained nurses. Red blood cell count, white blood cell count, absolute number of lymphocytes, and absolute number of neutrophils were measured using Sysmex XN9000 (Sysmex, Japan). C-reactive protein level was evaluated by the nephelometry immunoassay using the BN ProSpec System (Siemens, Germany).

### 2.5. Job Burnout and Job Stress

Job burnout in nurses was assessed using the Maslach Burnout Inventory (MBI) before and after the intervention. MBI was compiled by Maslach and Jackson in 1986 [20, 21] and translated in 2000 by Li. MBI has been shown to have good reliability and validity in the Chinese population [22]. Briefly, the MBI consists of 22 items in three dimensions: emotional exhaustion (nine items), depersonalization (five items), and reduced personal accomplishment (eight items). The nurses responded to each item using a 7-point Likert scale. The higher the score, the higher the degree of emotional exhaustion and depersonalization and the lower the degree of reduced personal accomplishments.

Job stress in nurses was evaluated using the China Nurses' Job Stressors Scale (CNSS) before and after intervention, which was compiled by Li in 1999 [22]. Briefly, the CNSS consists of 35 items in five dimensions: nursing specialty and work (seven items), workload and time allocation (five items), working environment and resources (three items), patient care (11 items), management, and interpersonal relationship (nine items). The nurses responded to each item using a 4-point Likert scale. The total score was between 35 and 140 with higher scores indicating higher levels of job stressors.

### 2.6. Statistical Analyses

G∗Power 3.1 software was used for sample size estimation. Based on our pilot results, a minimal sample size of 82 was suggested to reach a power of 0.80% and a significance of 0.05. Statistical analysis was performed using IBM SPSS Statistics software (version 22.0, IBM Corporation, USA). Numerical variables are expressed as the means and standard deviations (SDs) if data were normally distributed. Discrete data were expressed as frequencies or percentages. Differences between two groups were tested using the independent *t*-test and chi-squared test for continuous data and discrete data, respectively. Fisher's exact test was used in the analysis of contingency tables. A *P* value less than 0.05 was considered statistically significant.

## 3. Results

### 3.1. Baseline Information

A total of 185 patients participated in the study. Six patients were transferred to the intensive care unit due to severe postoperative cardiopulmonary disease and thus were excluded. The mean age of the participants was 63.6 years (SD = 7.3 years, range = 45–82 years). The ratio for female and for married was 76.5% and 96.6 %, respectively. Demographic and disease-related data of the participants are summarized in Table 2. Difference in these demographic and disease-related variables between two groups was not statistically significant (Table 2).

### 3.2. Postoperative Recovery and Complications

The hospitalization time and time to first ambulation, straight leg raising, and knee flexion to 90 degrees after the intervention in the video-assisted health education group were significantly shortened compared to those in the oral education group with data summarized in Table 3.

After the intervention, constipation and postoperative orthostatic intolerance were significantly reduced. Comparisons of postoperative complications are summarized in Table 4. The difference in the DVT rate between two groups was not statistically significant (*P* = 0.243).

### 3.3. Biomarkers

Levels of biomarkers are summarized in Table 5. CRP levels were significantly lower, and red blood cell counts were significantly higher in the intervention group when compared with the control group (*P* = 0.004 and *P* = 0.016, respectively).

### 3.4. Job Burnout and Job Stress in Nurses

Job burnout and job stress in nurses are summarized in Table 6. There were significant differences in emotional exhaustion, reduced personal accomplishments, and job stress between the two groups (*P* = 0.002, *P* = 0.004, and *P* < 0.001, respectively).

## 4. Discussion

In this study, video-assisted health education was shown to be more useful than oral education in promoting postoperative recovery on TKA patients and reducing job burnout and job stress in nurses.

Manpower shortage of nurse in the public healthcare system remains challenging, and thus, the registered nurses are under a heavy workload, which probably affects the quality of healthcare service. For example, in one survey, 51.6% of nurses believed that the main factor affecting nurses' performance of health education duties was time tension [23]. Furthermore, the heavy workload and differences in interpersonal communication skills, work efficiency, and personality of nurses were suggested to be the difficulties to achieve consistency, continuity, and standardization in patient education [24]. Therefore, an effective method by which nurses can maintain the quality of patient education in the situation of heavy workload is urgently warranted. Some clinicians suggested that using video health education has the potential to help patients memorize the information and reduce the workload of nurses at the same time [25]. The present study provided evidence for advantages of video-assisted health education over oral education in providing comprehensive, standardized, and easy-to-assimilate information, which accelerated postoperative recovery.

The condition of heavy workload increases the pressure of nurses. The application of video-assisted health education in the rehabilitation training on patients after TKA reduces repetitive explanation for questions that were commonly raised and for the inconsistent oral expressions. In this way, video-assisted health education can improve work efficiency of nurses and thus reduce their work pressure and job burnout. Besides, application of video-assisted health education can be extended to community care services, home care services, and other fields to promote rehabilitation training [26]. Health education assisted by a video could be at least a supplement to traditional teaching modes and standardize health education at relatively low cost in community.

Oxidative stress can cause oxidative damage to various macromolecules, and it has been considered to be one of the causative factors in the pathogenesis of KOA [2, 3]. TKA was demonstrated to be effective in reducing local chronic oxidative damage in OA patients [27]. Nevertheless, a level of oxidative stress continues during postoperative recovery until the peripheral tissues of the knee joint are repaired [28]. Video-assisted health education on rehabilitation training was found to be a macroscopic antistress strategy that modulated low-grade chronic inflammation and active antioxidant enzymes and stimulated the secretion of anti-inflammatory cytokines [12, 29]. Ihalainen and colleagues [30] reported a decrease in proinflammatory biomarkers, such as CRP and inhibited systemic or wound local inflammatory reactions after rehabilitation training. Chen and colleagues [31] suggested that active functional exercise after TKA improved the levels of TNF -*α*, IL-1*β*, and IL-6 and promoted the recovery of joint function. The present study enhanced the evidence for the benefits of rehabilitation training and further suggested an advantage of video-assisted health education over oral education in the training provided by nurses who had heavy workload.

This study has some limitations. First, confounding information about KOA classification and evaluation of knee function was not obtained, which may have led to bias in the results. Second, compliance of patients was not assessed, and it probably caused response bias, which may limit the generalizability of the study results. Therefore, further studies with confounding factors better controlled and with larger sample size are warranted.

## 5. Conclusion

Video-assisted health education may promote the recovery after total knee arthroplasty and reduce job burnout and job stress in nurses when compared with classical oral education. Video-assisted health education could be helpful in situation where manpower of nurse is in shortage.

## Figures and Tables

**Table 1:** Training after total knee arthroplasty.

Content	Method	Time
Ankle pump exercise	(i) Take supine position (ii) Actively flex and extend the ankle joint (iii) Relax the thigh (iv) Slowly and forcefully extend the ankle joint back as far as possible within the limit of no pain or only slight pain for 10 seconds (v) Plantar flexion for 10 seconds	5-10 minutes per hour

Intramuscular quadriceps isometric contraction exercise	(i) Take supine position with the knees straight (ii) Strain the thigh muscles for 5-10 seconds (iii) Relax and repeat	3-5 times per set, 10-20 sets per day
Hamstrings isometric contraction exercise	(i) Take supine position (ii) Press muscles in the posterior upper leg by extending the upper leg against pillows (iii) Relax and repeat	

Straight leg raising exercise	(i) Take supine position (ii) Hook up the toe of the affected limb (iii) Straighten and raise the leg to an angle of 30-40 degrees from the bed (iv) Maintain the position as long as possible (v) Relax and repeat	5-10 times per set, 3-5 sets per day

Flexion knee exercise in the supine position	(i) Take supine position (ii) The lower leg is relaxed and sagging naturally	5 minutes per set, 2-3 sets a day
Flexion knee exercise in the prone position	(i) Take prone position (ii) Flex the affected knee joint	

**Table 2:** Baseline information of the participants.

Variables	Intervention group (n = 91) (Mean ± SD)	Control group (n = 88) (Mean ± SD)	*t / χ* ^2^	*P* value
Age	62.87 ± 7.46	64.27 ± 7.20	-1.28	0.202
Gender				
Male	16	26	3.57	0.059
Female	75	62		
Marital status				
Single	3	3	0.002	0.967
Married	88	85		
Education				
Primary school and below	47	35	2.58	0.275
Junior middle school	25	29		
Senior high school and above	19	24		
Comorbidity				
Yes	58	57	0.021	0.885
No	33	31		
Pain score	2.34 ± 0.87	2.36 ± 0.94	-0.17	0.865
Barthel index score	89.67 ± 5.47	90.17 ± 5.59	-0.61	0.546

**Table 3:** Postoperative recovery of participants in the two groups.

Variables	Intervention group (n = 91) (Mean ± SD)	Control group (n = 88) (Mean ± SD)	*t*	*P* value
Hospitalization time (days)	7.51 ± 1.79	8.21 ± 2.15	-2.37	0.019
First ambulation (h)	19.91 ± 4.57	50.15 ± 7.00	-34.34	< 0.001
Straight leg raising (h)	26.55 ± 12.19	40.38 ± 11.64	-7.76	< 0.001
90 degrees flexion (h)	21.31 ± 5.83	35.72 ± 9.93	-11.88	< 0.001

**Table 4:** Complications in intervention and control groups.

Complications	Intervention group (*n* = 91)	Control group (*n* = 88)	*χ* ^2^	*P* value
DVT	10	15	1.37	0.243
Postoperative orthostatic intolerance	7	19	6.96	0.008
Constipation	10	23	6.83	0.009

**Table 5:** Count of blood cells in intervention and control groups.

Items	Intervention group (n = 91)		Control group (n = 88)		*t*	*P* value
	Mean ± SD	Coefficient of variation (%)	Mean ± SD	Coefficient of variation (%)		
CRP (mg/L)	84.54 ± 36.09	42.68	99.45 ± 31.73	31.90	-2.93	0.004
WBC (10^9^/L)	6.89 ± 1.60	23.16	7.38 ± 1.82	24.72	-1.90	0.060
RBC (10^12^/L)	3.73 ± 0.40	10.73	3.57 ± 0.46	12.77	2.44	0.016
LYMPH (10^9^/L)	1.33 ± 0.63	47.24	1.25 ± 0.42	33.76	1.04	0.300
NEUT (10^9^/L)	4.99 ± 2.98	59.69	5.40 ± 1.59	29.53	-1.15	0.254

CRP, C-reactive protein; WBC, white blood cell; RBC, red blood cell; LYMPH, absolute lymphocyte count; NEUT, absolute neutrophil count.

**Table 6:** Job burnout and job stress in nurses for intervention and control groups.

Items	Intervention group (n = 10) (Mean +/- SD)	Control group (n = 10) (Mean +/- SD)	*t*	*P* value
Emotional exhaustion	21.00 ± 8.04	36.50 ± 11.22	3.55	0.002
Depersonalization	9.10 ± 4.77	12.30 ± 7.53	1.14	0.271
Reduced personal accomplishments	41.90 ± 4.91	32.80 ± 7.07	-3.34	0.004
Job stress	55.90 ± 11.57	85.50 ± 6.80	6.97	<0.001

## Data Availability

Data are available from Shuang Wang (wangshuang200803@163.com) for researchers who meet the criteria for access to confidential data.

## Supplementary Materials

Supplementary Materials CONSORT 2010 checklist of information to include when reporting a randomised trial.
